The article "Detection of Pneumonia Infection by Using Deep Learning on a Mobile Platform" was published in 2022. Journal: Comput Intell Neurosci.

# Detection of Pneumonia Infection by Using Deep Learning on a Mobile Platform

**DOI:** 10.1155/2022/7925668

**Published:** 2022-07-30

**Authors:** Alhazmi Lamia, Alassery Fawaz

**Affiliations:** ^1^Department of Management Information System, College of Business Administration, Taif University, P.O Box 11099, Taif 21944, Saudi Arabia; ^2^Department of Computer Engineering, College of Computers and Information Technology, Taif University, P.O. Box 11099, Taif 21944, Saudi Arabia

## Abstract

Pneumonia is a disease that spreads quickly and poses a serious risk to the health and well-being of its victims. An accurate biomedical diagnosis of pneumonia necessitates the use of various diagnostic tools and the evaluation of various clinical features, all of which are hindered by the lack of available experts and tools. According to the research presented here, a mobile app that uses deep learning techniques to classify whether or not a patient has pneumonia is being developed. It was hoped that a mobile application prototype for detecting pneumonia using neural networks would be developed as part of this study. The use of a high-level tool such as Create ML makes this process easier and eliminates issues such as how many layers a neural network has, initializing the model parameters, or which algorithms to use. The model can now be accessed by anyone, anywhere, via a mobile application. The dataset of more than 5,000 real images was used to train an image classification model using Create ML, a tool with a graphical interface, and there was no need for specialized knowledge.

## 1. Introduction

In health services in Iraq, respiratory infections represent between 50 and 70% of consultations and between 30 and 60% of hospitalizations [1]. Among adults suffering from pneumonia, it is estimated that between 22 and 42% require hospitalization and between 5 and 10% need an intensive care unit, and the lethality varies between 5 and 50% depending on the severity of the condition, which is higher in the elderly and immunosuppressed patients [2–4].

The diagnosis of pneumonia requires a review of chest radiography (CXR) by a highly qualified specialist, laboratory tests, vital signs, and clinical history, which makes its detection a difficult task. It normally presents as an area of increased opacity within the CXR. Even so, the identification of the diagnosis of pneumonia is complex due to other pulmonary conditions such as hemorrhages, lung cancer, postsurgical changes, pulmonary edema, atelectasis, or collapse. The comparison of CRX performed at different times and the relationship with the clinical history is essential for diagnosis.

Taking advantage of the large number of images generated by digital processing [3], some studies [5–9] focus on methods based on convolutional neural networks (CNN) to define whether a patient has pneumonia or not since they learn and select functions automatically. Other works [10–13] highlight the analysis of cracks using artificial neural networks, hidden Markov model, modeling of Gaussian mixtures (Gaussian Mixture Models, GMM), and algorithm K-NN (K-Nearest Neighbors). Although the models that currently exist have achieved performances that rival expert doctors [14–16], these proposals mostly remain in algorithms or platforms and do not develop useful tools. Due to advances in machine learning and greater power in smartphones, some authors leave open the possibility of incorporating these algorithms, which in turn can generate a great demand for this type of tool [4].

This work seeks to design a mobile application for the automatic detection of pneumonia, which may be appropriate in regions where health professionals do not arrive or as support when defining a diagnosis to reduce the mortality rate associated with Pneumonia [17–20].

In this article, we present a prototype application for the support of medical personnel in the diagnosis of pneumonia through radiographic images of the patient's chest through the use of neural networks.

## 2. Theory

In this work, we present an application prototype to support medical personnel in the diagnosis of pneumonia through radiographic images of the patient's chest through the use of neural networks.

### 2.1. Pneumonia

Pneumonia is a form of acute respiratory infection that impacts the lungs, which are composed of alveoli that are small sacs. When healthy people breathe, their lungs should be allowed to fill with air [21]. People who have pneumonia have alveoli that fill with pus and fluid, which makes breathing painful and limits the amount of oxygen that can be absorbed. Pneumonia is the single most important contributor to infant mortality around the world.

### 2.2. Diagnosis of Pneumonia

It is detected from an interrogation or physical examination, where the doctor listens to the lungs with the help of a stethoscope to identify crackling, bubbling, whistling, and rumbling sounds when inhaling and exhaling.

To make an accurate diagnosis, it is recommended to carry out some tests, which can be chest X-ray, pleural fluid culture, pulse oximetry, blood oxygen measurement, and bronchoscopy.

### 2.3. Machine Learning

Automatic learning (Machine Learning) seeks to create techniques or systems that learn automatically, and through patterns, it analyzes and treats information. Once the patterns are identified, they are able to predict behaviors and continuously improve.

A task in machine learning known as supervised learning involves inferring a function from training data that has been labeled. In order to solve a problem that involves this learning, the following steps need to be followed in the correct order: determine the type of training example, assemble a training set, determine the input features, determine the structure of the learned function and the corresponding learning algorithm, finish the design, and evaluate the accuracy of the learned function.

Finding a hidden structure in data that does not have labels is the goal of unsupervised learning, which occurs when there is neither an error signal nor a reward with which to evaluate a potential solution. Methods such as clustering and latent variable models (including the expectation maximization (EM) algorithm, method of moments, and blind signal separation techniques) are examples of approaches to unsupervised learning. [22–25].

### 2.4. Artificial Neural Network (ANN)

They are computer systems [26–29] that try to emulate some of the functions of living organisms. This means that they are made up of elements that mimic (in basic functions) the behavior and organization of the organism. The human brain can learn from experience and generalize from previous input to completely new input to predict an outcome. A neural network gains experience by analyzing data (Training) to determine behavior rules [30–32], based on which it can make predictions about new cases.

### 2.5. Deep Learning

It is an area within the field of machine learning that brings together a set of algorithms and techniques; with this method, learning is sought through examples, obtaining patterns from large amounts of data [20]. In this technique, the artificial network of neurons is composed of several layers of processing in a hierarchical manner, each one from a lower level of abstraction to a higher one (inspired by the biological behavior of the brain by the interconnections between neurons), and each one of them with a task. Specifically, various architectures organize the connections of different layers to determine the direction and propagation of data. Convolutional networks, in particular, have quickly become a methodology of choice for image analysis.

### 2.6. Convolutional Neural Network (CNN)

It is a type of neural network specialized in the classification of images, videos, sounds, or text; its structure is similar to the visual cortex of a biological brain, so they are especially useful in locating patterns in images, recognizing objects, faces and scenes, and are widely used in the field of artificial division.

### 2.7. Review of the Literature

In 2018, Jakovljevic carried out a study on the tools to help diagnose pneumonia, where the focus is given on the analysis of the signals coming from the human body based on audio: cough, breathing, and speech, for the said signals. Starting from the common method, such as auscultation, the generated signal is processed with digital treatment techniques to be displayed, stored, and reproduced. This information must be processed to filter and eliminate noise and distortion so that it can be used as a training database. Among the studies, the analysis of crackles (discontinuous sounds of short duration) stands out using artificial neural networks, the Hidden Markov Model, Gaussian Mixture Modeling (GMM), and K-NN Algorithm (K-Nearest Neighbors), where it is concluded that neural networks and the K-NN algorithm give the best results in terms of monitoring respiratory sounds. It leaves open the possibility of introducing algorithms in increasingly powerful smartphones [33].

By 2019, Medrano Roldán using Apache Spark analyzed data as a framework in memory based on distributed processing and establishes how to implement a convolutional neural network to automatically classify radiographs of patients with pneumonia as the database that is stored increases. The analyzes concluded that the database contains “x-rays of patients with pneumonia regardless of whether it is due to viruses or bacteria, and patients with a normal diagnosis where it is finally reduced to two classes, with and without pneumonia.” She divided into 10 data sets, reduced the total number of images from 5,856 to 3,166 to avoid an imbalance, and normalized the images by training and evaluating the network with each data set [12, 13].

Also, in 2019, Samir Yadav and Shivajirao Jadhav [14] compared studies where images are used to diagnose diseases, where they highlighted the implementation of deep neural networks (DNN), especially convolutional neural networks (CNN), and achieved significant performance since 2012. They show that some investigations on the classification of medical images by CNN have managed to rival human experts. Where they give us an example CheXNet, a CNN with 121 layers trained with more than 100,000 frontal view chest X-rays, obtained better performance than the average performance of four radiologists. He further states that Kermany proposes a transfer learning system to classify images where the weighted average error is equal to the average of 6 human experts.

Abate (2019) et al. [15] mentioned significant achievements of CNNs in large amounts of data sets, but for cases where the data set is small, it sometimes fails if proper care is not taken. They propose a transfer learning approach using pretrained architectures to obtain the same result between small and large ensembles. They used five pretrained models, where they took the combination of them to form a large ensemble architecture and achieved promising results.

From the previous works, we can conclude that the approach that has been given by different researchers over time has been aimed at establishing algorithms that can select the characteristics automatically and evaluations to reduce false positives when classifying the diagnosis of pneumonia, but none has made an application on a mobile device as a support tool for the detection of pneumonia.

## 3. Methodology Implementation

The project is developed under the CRISP-DM methodology [16] used for development projects in the area of Data Analytics; it describes the common activities that must be carried out for the completion of a project of this nature; it consists of the next six phases.

### 3.1. Business Understanding

In this phase, the business objectives and current needs are determined. For this, it is necessary to carry out a review of the current technologies in the diagnosis of pneumonia, the actors, time, and availability not only for medical personnel but for the general public; with this information, the development is proposed and limited to the project.

### 3.2. Understanding the Data

The data collection process is carried out by searching different sources of information. The data used for the creation of our model was obtained from http://www.cell.com/cell/fulltext/S0092-8674(18)30154-5. These contain images of chest radiographs in patients with pneumonia of different causes and healthy patients.

### 3.3. Preparation of Existing Data

To carry out the training, it is necessary to have a data set organized and classified in these two categories; it is also important to have a group of data for training and another set for tests. It is not recommended to use training data to carry out tests, but it is recommended to use 80% of data for training and 20% for testing. At least 10 images are required for each category (NORMAL and PNEUMONIA). The more data there is, the better the accuracy of the model; the number of images in each category must be balanced as far as possible; 10 images cannot be used in the NORMAL category and 1,000 images in the PNEUMONIA category.

The images can be in any jpeg, png, or other formats (Figure 1); the images do not have to be the same size or have a specific size. However, it is better to use images of at least 299 × 299 pixels.

### 3.4. Modeling

For modeling, Create ML is used. For several years, Apple has been venturing into the world of machine learning and also offering tools so that developers can easily integrate these features into applications. In this way, at WWDC, I present the Create ML, an application to build, train, and implement machine learning models directly from a Mac, without the need for Internet and advanced knowledge in machine learning [17–21].

Create ML (Figure 2) is a new way to train custom machine learning models that offers a simple and intuitive interface generating an extremely simplified experience; you can train models to perform tasks such as recognizing images, extracting meaning from text, or finding relationships between numerical values, all it requires is a sufficient amount of data for training.

Create ML Takes advantage of the machine learning infrastructure integrated into Apple products such as Photos and Siri, among other frameworks that come directly with the device; this makes some models smaller, more efficient, and require much less training time.

Currently, there are other very popular tools for creating custom models, such as Tensorflow and Caffe, but these require a large amount of code and do not have a friendly interface, and often require command of a programming language such as Python and some libraries. There are also other cloud-focused tools like Google Cloud AutoML and IBM AutoAI, but these require a constant Internet connection for data loading and training.

In the case of Google Cloud AutoML and Create ML, the difference between the accuracy of the models obtained using these two tools is not significant; both tools are good enough, and the decision on which to choose depends on personal preferences, availability of Internet, equipment, and storage space.

Create ML accepts various input types available for creating models images, sound, text, and number tables. In this case, a model will be used that uses an image as input and classifies it into two categories according to its content, NORMAL and PNEUMONIA.

#### 3.4.1. Model Type Selection

To train a model using Create ML, it is necessary to create a project based on the different model templates; these are grouped according to the type of input of the model that we want to train.

After selecting “Image Classifier, “Select” Next”, and we put some complementary data such as the name of the project, license, description of the model, and location of the project. Then the main interface is shown, which is quite simple and intuitive; you can train multiple versions of the same model using different datasets simultaneously. In the left panel, the different resources of the model are shown, and in the right panel, the data flow goes from left to right with the steps required to perform in the training, from inputting data to finishing with the output of the trained model (Figure 3(a)).

#### 3.4.2. Entry

The input data for model training is divided into three groups:

1. Training: classified data that the model will use to learn
2. Validation: data that the model will use to verify the learning in each iteration, the application allows to take them randomly from the training set
3. Tests: for the data that the application will use to verify the model's efficiency, it is important that none of these images are in the training set

To select the data, it is only necessary to drag and drop the folder with the images in the corresponding section.

Additionally, some options are allowed to be configured, such as the maximum number of iterations for the training and some filters that will be applied to each image to increase the amount of data when there is not a good number of data, and you want to improve model accuracy.

#### 3.4.3. Training

Once the different data sets have been selected and the parameters configured, you can start training the model; you only need to press the “Training” button located on the toolbar (Figure 3(b)), and you can see the progress live as the model learns from the training images.

The model learning process is iterative; in each iteration, the model learns according to the characteristics of the training data set and verifies the accuracy with the validation data set because the validation data is generated randomly. The model may vary each time the model is trained.

The training time depends on factors such as the amount of data, number of iterations, filters applied to each image, and the team's capabilities.

#### 3.4.4. Assessing Model Accuracy

Once the training is complete, you will be able to see different metrics of this process; creating ML shows the precision values with the training and validation data; this gives us information on how well the model is trained and allows us to make decisions.

The accuracy value for the training dataset is always close to 100% because the model has trained on these images. In our case, the model correctly identified 97% of the validation images and 86% of the test images.

The application also shows additional information on the training progress in each iteration, such as the number of elements in each category, precision, number of iterations, and total training time (Figure 4(a)).

Create ML to check the efficiency of the trained model against the test dataset, which contains images that the model has never seen before.

The model classifies all the images, and the app compares them to the correct category and presents the overall accuracy. For the first training, a general accuracy of 86% was obtained, and the accuracy for each category NORMAL (Healthy) 90% and PNEUMONIA 84% can also be observed; this indicates how good the model is to hit in each category (Figure 4(b)).

Suppose the performance of the model is very low, in that case, another training can be carried out with different parameters, increasing the number of iterations or with another more varied set of data, for example, images with different light exposures. This process can be carried out as many times as necessary to obtain the expected results. Create ML allows multiple training sessions to be carried out on the same model with different configurations and to compare the results of each of them in the same project. In this case, it can be seen that the performance can worsen depending on the parameterization (Figure 5(a)).

#### 3.4.5. Exporting the Model

In the “output” section, the application allows testing with multiple images and shows the results of the classification (Figure 5(b)). When it is determined that the model works well enough, you can save the trained model to use; it is only necessary to drag and drop the model outside the application. It generates a file with the.mlmodel format, which is ready to be used in any application in the Apple ecosystem (iOS, iPadOS, macOS). One of the benefits of using Create ML to build models is how extremely small they are, and in this case, the model is only 17 KB.

### 3.5. Evaluation

Validation is performed according to expert judgment using the graphs obtained from the model accuracy training process to the group of test and validation images. At this point, it was possible to determine that the model is useful according to the needs of the business and meets the objectives to continue with the application prototype.

### 3.6. Implementation

Building the classification model by itself is not useful if it is not integrated into some application or service that uses it. This is why it is determined that a simple way to implement the model is through a mobile application; interested people can easily access it and use the device to capture or upload radiographic images for the model to make the prediction. The SCRUM methodology [34] is used to develop the application prototype.

Integrating pneumonia.mlmodel model in an iOS application is quite simple since the entire Apple ecosystem provides the tools to make this process as simple as possible; it can be used with a few lines of code.

Xcode is the integrated development environment offered by Apple for building applications. To use the model, it is only necessary to drag the model to a project in Xcode. Once the model is part of the project, Xcode displays the model information, type, description, size, input, and output data.

Thanks to the different frameworks included in Xcode, such as Core ML and Vision, classes are automatically created for the use of the model; other frameworks such as AVFoundation and PhotoKit allow us to obtain the images that are used as input for the model, whether they are from the device's camera or the photo library. Only a few lines are required to use the model in code, with which classification and a confidence percentage of this prediction are obtained from an image.

### 3.7. Functioning of the Application Prototype

The application consists of a few simple steps; the user can use the camera to take a photo or import a certain image from the photo gallery for analysis; once the user selects the image, the application processes it and displays the result with the prediction and the percentage of confidence offered by that result. The following are screenshots of the app on an iPhone 11 emulator, as shown in (Figure 6).

## 4. Results and Discussion

Data is the most important part of the project, and having a sufficient and reliable data set is the key to success. Performing the training of an image classifier model through the CreateML application is simple; unlike other tools, it abstracts the entire process in a simple interface, which means that great knowledge is not required to carry out the said process. The application allows the configuration of parameters and multiple workouts with different configurations; it generates graphs that allow us to make decisions, as shown in (Figure 7).

The classification models are composed of multiple layers in charge of carrying out simple processes and communicating these results to other layers to classify an image. The first layers are responsible for taking the raw pixel values and generating high-level abstract ideas such as “it's white” or “it's an animal” as you move between layers, and more specific details of the images are obtained until you can distinguish between NORMAL and PNEUMONIA (Figure 8). There are also different ways to organize and communicate the different layers and there are different architectures to organize these layers depending on the type of problem to be solved. Still, all this process is internal, thanks to CreateML.

After carrying out several training processes with different configurations and variations in the parameters, it was possible to obtain a model with an accuracy of ∼85% integrated into an iPhone application that is very easy to use and distribute.

Since the model was trained with a set of data closed to two categories, NORMAL (Healthy) and PNEUMONIA, any image passed as input to the model will be categorized into one of these two groups since, during the training process.

If the image of a cat is sent, the model will respond incorrectly with the label PNEUMONIA. To solve this problem, you can choose to create another category of training data called OTHERS. It contains various images of things or objects that the user could pass as input to the model *to* improve the user experience.

It was also possible to show that factors such as lighting, contrast, blur, shooting angle, background, and different distortions present in the input image can affect the model's accuracy because within the training group, they are not being considered. Example images are those with these factors so that the model learns these characteristics with these variations. It is enough to include images of this type in the different data sets to solve this problem. The images present in the training process should be as close as possible to what is expected as input to the model, that is, how the end-user is expected to take the images.

## 5. Conclusions and Recommendations

### 5.1. Conclusions

The objective of this research work was to propose a mobile application prototype for the detection of pneumonia from a chest X-ray image through the use of neural networks. The model was created using Create ML, a high-level tool that simplifies this process and eliminates challenges, such as choosing how many layers a neural network has, initializing the model parameters, or what algorithms to use. The implementation of the model in a mobile application offers its use to anyone; the source code of the application is available on Github.

It was possible to establish through the review of the state of the art that there are various investigations to address the diagnosis of pneumonia using the field of artificial intelligence; some of them use radiographic image analysis and others stand out for analysing lung sounds. Many of these research projects focus on enhancing the efficiency of the models and end with their training. No research was found that uses the potential of mobile devices for the deployment of these models, although some authors leave this possibility open. This research offers an approach to the said processes to fill this existing gap.

Although artificial intelligence has been talked about since the middle of the last century, the most important advances have been made in recent years with the improvement of technique and technology; these improvements have intensified its use in different fields such as image recognition, voice, stock prediction, text generation, language translation, fraud prevention, autonomous driving, genetic analysis, and disease prognosis, being in the field of medicine one of the most interesting as it can help both medical staff and patients to make quick and accurate decisions, thus being able to save lives by offering early treatment. Using the existing data, it was possible to train several models with different configurations whose accuracies vary between ∼78% and ∼85%; we can conclude that the model's capabilities can be expanded if sufficient training data is available.

The model that obtained the best results was implemented in a mobile application prototype. The device's camera or photo gallery can be used for the application to process and generate a forecast. Its use is quite simple and generates a good user experience, the size of the application is only 4.8 MB, and the response time using the model is less than 1 second.

Future work can use a richer and more varied data set to classify different types of lung diseases. It is also possible to analyze other types of images such as MRIs or mammograms to predict whether a patient is likely to develop cancer.

### 5.2. Recommendations

For future projects related to image analysis and classification, we recommended the following:

1. The data groups must be balanced in all the categories you want to classify
2. They must have the most examples for each category
3. The training data must fit the expected data as input to the model
4. Different environmental conditions, such as lighting, can affect the model results, so it is important to have images in different conditions in the training data

## Figures and Tables

**Figure 1:** Data structure.

**Figure 2:** Creating ML from Apple (https://developer.apple.com/documentation/createml).

**Figure 3:** (a) Configuring input data for model training and (b) model training.

**Figure 4:** (a) Training results; (b) model tests.

**Figure 5:** (a) Retraining results with different parameters, (b) training result and tests with the model.

**Figure 6:** Application operation in an iPhone 11 emulator.

**Figure 7:** Graph of training results of a model.

**Figure 8:** Classifier model training flow.

## Data Availability

The data used to support the findings of this study are included within the article.
